# Quantitative Identification of Antioxidant Basis for Dendrobium Nobile Flower by High Performance Liquid Chromatography-Tandem Mass Spectrometry

**DOI:** 10.1155/2022/9510598

**Published:** 2022-08-19

**Authors:** Dan Rao, Yadong Hu, Ruoxi Zhao, Hongjie Li, Ze Chun, Shigang Zheng

**Affiliations:** ^1^CAS Key Laboratory of Mountain Ecological Restoration and Bioresource Utilization & Ecological Restoration and Biodiversity Conservation Key Laboratory of Sichuan Province, Chengdu Institute of Biology, Chinese Academy of Sciences, Chengdu 610041, China; ^2^University of Chinese Academy of Sciences, Beijing 100041, China; ^3^Innovation Academy for Seed Design, Chinese Academy of Sciences, Beijing 100101, China; ^4^Xiongan Institute of Innovation, Chinese Academy of Sciences, Baoding 071000, China

## Abstract

*Dendrobium nobile* is a beautiful orchid and a widely used medicinal plant. In vitro antioxidant assays suggested that *D. noblie flower extracts* showed significantly higher 2, 2′-azinobis-3-ethylbenzthiazoline-6-sulfonate (ABTS) and 1, 1-diphenyl-2-picrylhydrazyl (DPPH) scavenging rates and much more ferric-reducing power than those of root, stem, leaf and fruit. To better understand the antioxidant basis of *D. nobile* flower, high-performance liquid chromatography tandem mass spectrometry (HPLC-MS/MS) was used for metabolic identification and quantification. Finally, there were 72 metabolites among the total of 712 identified components showed significant association (coefficient >0.8, *p* < 0.05) with ABTS scavenging rates, DPPH scavenging rates, and ferric-reducing power. The three enriched classes of flower metabolites, including amino acids and their derivatives, organic acids and their derivatives, and flavonoids, formed the main antioxidant basis. The significantly accumulated rutin, astragalin, isomucronulatol-7-O-glucoside, quercetin 4′-O-glucoside, methylquercetin O-hexoside, caffeic acid, caffeic acid O-glucoside, and *p*-coumaric acid (Log_2_(fold change) >2, *p* < 0.01, distribution in flower >0.1%) made a key contribution to the higher antioxidant activities in flower. The relative quantification results of HPLC-MS/MS were verified by the common quantification methods. The antioxidant basis revealed of *D. nobile* flower will be helpful in the production of healthy or beauty products.

## 1. Introduction

*Dendrobium nobile* Lindl. is one of the endangered orchids, which has been used as a medicinal plant for many years in China, Japan, India, and some other countries [1, 2]. It showed many health beneficial functions, such as eye-protection, liver-protection, cardiovascular-protection, gastric-protection and neuro-protection [3, 4].

Oxidative stress is associated with the occurrence and progression of cancer, metabolic syndrome, diabetes, cardiovascular disease, hypertension, Alzheimer's disease, and aging [5–7]. Thus, antioxidant activities attached more and more attentions in production of health-care foods or skin-care products [8]. Recent research indicated that some *Dendrobium* species might be good antioxidant resources. The reports on *D. officinale*, *D. chrysanthum*, *D. speciosum*, *D. chrysotoxum*, *D. denneanum*, *D. crepidatum*, *D. densiflorum*, *D. huoshanense*, *D. macrostachyum*, *D. signatum*, *D. catenatum*, *D. moniliforme*, *D. thyrsiflorum*, *D. fimbriatum*, *D. pachyglossum*, *D. aphyllum*, *D. devonianum*, and *D. sabin* showed that they performed effects on 1, 1-diphenyl-2-picrylhydrazyl (DPPH) scavenging, 2, 2′-Azinobis-3-ethylbenzthiazoline-6-sulphonate (ABTS) scavenging, or ferric reducing [9–14].

However, there were poor researches reported on the antioxidant basis of *Dendrobium* [8, 15]. In plant secondary metabolites, flavonoids, phenols, vitamins, organic acids, and polysaccharides are well known as good antioxidants [16–18]. Some flavonoids, such as quercetin, rutin, and isoquercitrin, had been reported to be correlated antioxidant activities in *D. officinale*, *D. catenatum*, and *D. huoshanense* [12, 19–21]. Some polysaccharides were also considered as functional antioxidants in *D. officinale*, *D. huoshanense*, and *D. nobile* [15, 22, 23]. Recently, high performance liquid chromatography-tandem mass spectrometry (HPLC-MS/MS) had been used for metabolic analysis, chemical differentiation, quality control, and pharmaceutical identification in some *Dendrobium* species [19, 20, 24]. This is helpful for further quantitative identification of some novel antioxidants in *D. nobile*.

The in-vitro antioxidant activities of the extracts from different tissues of *D. nobile* will be firstly evaluated in this paper. HPLC-MS/MS is then employed for metabolic analysis. The final co-analysis will indicate the main chemical basis for the respective antioxidant activities.

## 2. Materials and Methods

### 2.1. Plant Materials

Fresh roots, stems, leaves, flowers, and fruits of *D. nobile* were obtained from Hejiang, Sichuan Province (28°49′N, 105°50′E). Roots, stems, leaves, and flowers were collected in May 2019 and May 2020, fruits were collected in November 2019 and November 2020. Tissue samples were obtained from more than 30 individual plants for each collection. The tissue samples were washed with pure water, dried at 40°C for a week, ground into powder, and screened with a 50 mesh sieve before extraction.

### 2.2. Chemical Reagents

DPPH and ABTS were purchased from Beijing Zhongsheng Ruitai and Shanghai Macklin (China). The methanol, formic acid, potassium ferrocyanide, ferric chloride, and citric acid standard were purchased from Chengdu Kelon (China). The quantitative BCA protein kit and the bovine serum albumin (BSA) standard were purchased from Beijing Solarbio (China). The Rutin Standard was purchased from Chengdu Purechem-Standard (China).

### 2.3. Metabolites Extraction for Bioactivity Analysis

Each 5 g fine powdered sample was immersed with 200 mL of solution (80% methanol contained 0.1% formic acid) at room temperature for 24 hrs, and then was paper filtered to remove the residues. Subsequently, the filtrates were condensed in a rotary evaporator at 40°C for 2 hrs, and then were evaporated under vacuum for final drying. The dry extracts were dissolved with 80% methanol that contained 0.1% formic acid at a final concentration of 100, 200, 500, 1000, and 2000 *μ*g/mL for in vitro analysis.

### 2.4. DPPH Scavenging Assay

Each 0.3 mL extract was mixed with 0.9 mL methanol containing 0.1 mM DPPH. The mixed solution was kept at room temperature in the dark for 30 min before measuring the absorbance at 517 nm. The DPPH scavenging activity was calculated as follows: DPPH scavenging activity (%) = (*A*_0_ − *A*_*s*_)/*A*_0_ *∗* 100% (*A*_0_ absorbance without sample; *A*_*s*_ absorbance with sample). Vitamin C was used as a positive control [12].

### 2.5. ABTS Scavenging Assay

ABTS was dissolved in 0.01 M PBS at a final concentration of 7 mM (pH 7.4). The ABTS solution was reacted with 2.45 mM potassium persulfate at room temperature for 16 hrs without light to generate free radicals. Before use, the ABTS solution was diluted with 0.01 M PBS to an absorbance of 0.7 at 734 nm. Each 0.1 mL extract was mixed with 1 mL diluted ABTS solution. The mixed solution was kept at room temperature for 20 min before measuring absorbance at 734 nm. The ABTS scavenging activity was calculated as follows: ABTS scavenging activity (%) = (*A*_0_ − *A*_*s*_)/*A*_0_ *∗* 100% (*A*_0_ absorbance without sample; *A*_*s*_ absorbance with sample). Vitamin C was used as a positive control [9].

### 2.6. Ferric Reducing Assay

Each 0.1 mL extract was mixed with 0.5 mL 0.2 M PBS (pH 6.6) and 0.5 mL potassium ferrocyanide (K_3_Fe(CN)_6_, 30 mM). The mixed solution was incubated at 50°C for 20 min before addition of 0.5 mL trichloroacetic acid (0.6 M). Then, 0.5 mL mixed solution was further added with 0.5 mL deionized water and 0.1 mL ferric chloride (FeCl_3_, 6 mM). The absorbance was measured at 700 nm. The ferric reducing antioxidant power is calculated as follows: reduce capacity = *A*_*s*_ − *A*_0_ (*A*_0_ absorbance without sample; *A*_*s*_ absorbance with sample). Vitamin C was used as a positive control [13].

### 2.7. Metabolites Extraction for HPLC-MS/MS

Each 100 mg fine powdered sample was suspended with a pre-chilled 500 *μ*L solution (80% methanol contained 0.1% formic acid) by well vortex. The sample was incubated for 5 min and then centrifuged at 12,000*g* for 10 min. The supernatant was diluted to a final concentration of 53% methanol by pure water. The sample was then transferred to a new tube and then centrifuged at 12,000*g* for 20 min. The supernatant was used for chromatography.

### 2.8. HPLC-MS/MS Analysis

HPLC-MS/MS analysis were performed using an ExionLC™ AD system (SCIEX, USA) coupled with a QTRAP® 6500+ mass spectrometer (SCIEX, USA) in Novogene Co., Ltd. (Beijing, China). For positive ion mode, the sample was injected into a BEH C8 column (100 × 2.1 mm, 1.9 *μ*m) using a 30-min linear gradient at a flow rate of 0.35 mL/min. The eluents were eluent A (0.1% formic acid-water) and eluent B (0.1% formic acid-acetonitrile). The solvent gradient was set as follows: 5% B, 1 min; 5%–100% B, 24.0 min; 100% B, 28.0 min; 100%–5% B, 28.1 min; 5% B, 30 min. For negative ion mode, sample was injected into a HSS-T3 Column (100 mm × 2.1 mm) using a 25 min linear gradient at a flow rate of 0.35 mL/min. The eluents were eluent *A* (0.1% formic acid-water) and eluent *B* (0.1% formic acid-acetonitrile). The solvent gradient was set as follows: 2% *B*, 1 min; 2%–100% *B*, 18.0 min; 100% *B*, 22.0 min; 100%–5% *B*, 22.1 min; 5% *B*, 25 min. The mass spectrometer was operated in positive or negative polarity mode with curtain gas of 35 psi, medium collision gas, ion spray voltage of 5500 V or −4500 V, temperature of 500°C, ion source gas of 1 : 55, ion source gas of 2 : 55.

### 2.9. Identification and Quantification of Metabolic Molecules

The data files generated by HPLC-MS/MS were processed using SCIEX OS version 1.4 to integrate and correct the peak. The main parameters were set as minimum peak height of 500, signal/noise ratio of 5, and gaussian smooth width of 1. Each peak of the experimental samples was detected using multireaction monitoring (MRM) based on the Beijing Novogene internal database (China). The parent ion (Q1), the daughter ion (Q3), the retention times (RTs), the de-clustering potential (DP), the collision energy (CE), and the molecular weights (MWs) were used for the identification of the metabolites. The peak area of Q3 was used for relative quantification of the metabolites. These metabolites were further annotated using the KEGG database (https://www.genome.jp/kegg/), the HMDB database (https://www.hmdb.ca/), and the Lipidmaps database (https://www.lipidmaps.org/).

### 2.10. Detection of Total Flavonoids

Each 0.25 g fine powdered sample was added with 4 mL of 80% methanol in a 10 mL centrifuge tube. After ultrasonic extraction for 30 min and centrifugation at 9,000*g* for 10 min (4°C), the supernatant was collected. The residue was extracted with 4 mL of 80% methanol once-more. The combined supernatant was fixed to 10 mL with methanol. Each of 0.5 mL sample solution was mixed with 0.15 mL 5% sodium nitrite solution for 6 min. They were mixed with 0.15 mL 10% aluminum nitrate solution for 6 min. They were further mixed with 2 mL 4% sodium hydroxide solution and 2.2 mL distilled water for 3 min. The absorbance was determined at 508 nm and the total flavonoid content was calculated with the rutin standard.

### 2.11. Detection of Total Proteins

Each 0.1 g fine powdered sample was extracted with 1 mL 0.05 mM PBS (pH 7.8) by shaking for 2 hrs at room temperature. Then, each 20 *μ*L of the extracted filtrate was added with 200 *μ*L of BCA working solution (50 : 1 of bicinchoninic acid and Cu reagent). After mixing well, they were placed at 37°C for 30 min. The absorbance at 562 nm was used for calculation of total proteins with BSA standard.

### 2.12. Detection of Total Organic Acids

Each 0.25 g fine powdered sample was extracted with 100 mL of distilled water by shaking for 3 hrs at room temperature. Accurately take 50 mL of the extracted filtrate into a 250 mL beaker. Then, basic burette filled with sodium hydroxide solution was used for titration. The end point of the titration was pH 7.0. Citric acid standard was used for calculation. Organic acid content = (*C* *∗* *V* *∗* *M*)/(3 *∗* m) *∗* 100% (C concentration of sodium hydroxide solution; *V* volume of sodium hydroxide solution consumed by titration; *M* mass of citric acid; *m* mass of sample).

### 2.13. Statistics Analysis

All measurements and experiments were repeated at least three times. Quantitative data were presented as mean ± standard deviation (SD). The correlation analysis was performed using PASW statistics 18.0 (IBM, USA). Pearson correlation coefficients and *p* value were used for evaluating the correlations. Student's *t*-test was used for comparison between two groups. Log_2_ (fold change) was used for comparison of relative quantification. CSCF/TCCF (ratio of the contents of one specific component in flower to the total contents of all components in flower) and CSCF/CSCA (ratio of the contents of one specific component in flower to the contents of this component in all of root, stem, leaf, flower, and fruit) were used for comparison of different distributions.

## 3. Results and Discussions

### 3.1. Relatively Higher Antioxidant Activities Showed by Extracts of D. Nobile Flower

The ABTS and DPPH scavenging rates and ferric-reducing power of the extracts from root, stem, leaf, flower, and fruit increased in a concentration-dependent manner (Figure 1). Under the concentration of 100, 200, and 500 *μ*g/mL, the ABTS scavenging rates of flower extracts were significantly higher than those of extracts from root, stem, leaf, and fruit (*p* < 0.01). Under the concentration of 100, 200, 500, and 1000 *μ*g/mL, the DPPH scavenging rates of flower extracts were significantly higher than those of extracts from root, stem, leaf, and fruit (*p* < 0.05). At a concentration of 500, 1000, and 2000 *μ*g/mL, the ferric-reducing power of flower extracts was significantly higher than those of extracts from root, stem, leaf, and fruit (*p* < 0.05). When the concentration was greater than 500 *μ*g/mL, the ABTS and DPPH scavenging rates of flower extracts were close to those of vitamin C. In summary, flower extracts showed higher ABTS and DPPH scavenging rates and much more ferric-reducing power than those extracts from other tissues. These results revealed relatively higher antioxidant activities in vitro in the *D. nobile* flower.

### 3.2. Distribution of Metabolites in the Flower of *D*. *nobile*

A total of 712 metabolites were identified in the flower of *D*. *nobile* by HPLC-MS/MS (Figure 2). The 712 metabolites were classified into 11 classes, including amino acids and their derivatives (123), flavonoids (111), organic acids and their derivatives (105), phenols (62), nucleotide and its derivatives (67), carbohydrates (56), lipids (34), terpenoids (33), alkaloids (30), phenylpropanoids (20), and others (71). Relative quantification based on the peak areas of each metabolite showed its distribution in the flower of *D*. *nobile* (Figure 3). The top four distributed classes were amino acid and its derivatives (35.23% of CSCF/TCCF), Carbohydrates (17.44% of CSCF/TCCF), organic acid and its derivatives (13.76% of CSCF/TCCF), and flavonoids (13.31% of CSCF/TCCF).

### 3.3. Enriched Metabolites in Flower of *D*. *nobile*

There were 46 metabolites that showed a significant enrichment in the flower of *D. nobile* (Log_2_(FC) >2, Figure 4). Among them, flavonoids like kaempferol, quercetin, cyanidin and their derivatives accounted for a large proportion, such as quercetin, rutin (quercetin 3-O-rutinoside), quercetin 3-*β*-D-glucoside, quercetin 4′-O-glucoside, quercetin 5-O-hexoside, quercetin O-malonylhexoside, quercetin-3′-O-glucoside, quercetin-O-glucoside, methyl-quercetin O-hexoside, astragalin (kaempferol-3-glucoside), kaempferol 3-O-glucoside-2′-O-rhamnoside, kaempferol7-O-*β*-D-glucopyranoside, trifolin (kaempferol-3-O-*β*-D-galactoside), tiliroside (kaempferol-3-*β*-D-6″-p-coumaroyl-glucopyranoside), cyanidin 3-O-glucoside, cyanidin O-acetylhexoside, cyanidin O-rutinoside. There were also some other amino acids and their derivatives such as methionine, and organic acids and their derivatives such as p-coumaric acid and caffeic acid showed relatively high distribution. More, the top five of them were quercetin 3-*β*-D-glucoside (2.72% of CSCF/TCCF, 86.61% of CSCF/CSCA), rutin (2.40% of CSCF/TCCF, 96.16% of CSCF/CSCA), quercetin-3′-O-glucoside (2.29% of CSCF/TCCF, 86.96% of CSCF/CSCA), myricitrin (1.38% of CSCF/TCCF, 85.96% of CSCF/CSCA), caffeic acid (1.33% of CSCF/TCCF, 98.91% of CSCF/CSCA).

### 3.4. Metabolites Associated with Antioxidant Activities in Flower of *D*. *nobile*

After correlation analysis, there were 72 metabolites showed significant association (coefficient >0.8, *p* < 0.05) with the ABTS and DPPH scavenging rates and ferric-reducing power (Table 1). As shown in Figure 5, the 72 metabolites were mainly belongs to three classes of amino acid and its derivatives (13, 60.45% of CSCF/TCCF), organic acid and its derivatives (11, 19.05% of CSCF/TCCF), flavonoids (20, 17.05% of CSCF/TCCF). The average CSCF/CSCA of amino acid and its derivatives, organic acid and its derivatives, and flavonoids were 55.05%, 67.42%, and 81.15%. Antioxidant activities associated with amino acids and their derivatives showed a higher distribution in the flower itself, but antioxidant activities associated with flavonoids showed a higher distribution in the flower compared to the root, stem, leaf, and fruit.

### 3.5. Antioxidant Basis of *D*. *nobile* Flower

Among the 13 antioxidant activities associated amino acid and its derivatives, L-leucine (37.86%), L-isoleucine (25.90%), D-glutamine (23.16%), and D-norvaline (10.97%) showed relatively high distribution in flower itself (Figure 6(a)). But none of them showed more than 80% of CSCF/CSCA (Figure 7(a)). Among the 11 antioxidant activities associated with organic acid and its derivatives, pipecolinic acid (50.43%), caffeic acid (20.79%), pipecolic acid (10.74%), p-coumaric acid (9.37%), and caffeic acid O-glucoside (5.11%) showed a relatively high distribution in the flower itself (Figure 6(b)). But only caffeic Acid, p-coumaric acid, and caffeic acid O-glucoside showed more than 80% of CSCF/CSCA (Figure 7(b)). Among the 20 antioxidant activities associated flavonoids, rutin (41.78%), astragalin (14.29%), isomucronulatol-7-O-glucoside (12.48%), quercetin 4′-O-glucoside (11.58%) and methylquercetin O-hexoside (7.26%) showed a relatively high distribution in the flower itself (Figure 6(c)). And all of them showed more than 80% of CSCF/CSCA (Figure 7(c)). The main classes of metabolites and key components contributed to antioxidant activities were summarized in Figure 8. They were the identified antioxidant basis of *D. nobile* flower.

### 3.6. Verification of the HPLC-MS/MS Results

Relative quantification by HPLC-MS/MS showed that the distributions of amino acids and their derivatives in root, stem, leaf, flower, and fruit were 7.39%, 10.57%, 25.44%, 45.74%, and 10.85%, respectively (Figure 9(a)). The BCA method showed that total protein concentrations in root, stem, leaf, flower, and fruit were 32.24 mg/g, 24.29 mg/g, 253.59 mg/g, 288.18 mg/g, and 92.09 mg/g, respectively (Figure 9(d)). Relative quantification by HPLC-MS/MS showed that the distributions of organic acid and its derivatives in root, stem, leaf, flower, and fruit were 13.81%, 10.54%, 21.56%, 25.02%, and 29.06%, respectively (Figure 9(b)). The titration method showed the concentrations of total organic acids in root, stem, leaf, flower, and fruit were 1.17 mg/g, 0.68 mg/g, 1.66 mg/g, 1.73 mg/g, and 2.33 mg/g, respectively (Figure 9(e)). Relative quantification by HPLC-MS/MS showed that the distributions of flavonoids in root, stem, leaf, flower, and fruit were 0.65%, 4.55%, 27.25%, 53.62%, and 13.94%, respectively (Figure 9(c)). The colorimetric method showed that total flavonoids concentrations in root, stem, leaf, flower, and fruit were 8.72 mg/g, 9.23 mg/g, 12.49 mg/g, 31.30 mg/g, and 11.91 mg/g, respectively (Figure 9(f)). These results indicate that the relative quantification by HPLC-MS/MS was consistent with absolute quantification by the corresponding common methods.

### 3.7. HPLC-MS/MS was Suitable for Metabolic Identification and Quantification in Chemical-Function Analysis

The metabolism of plant was hugely complex. The high-throughput property of HPLC-MS/MS makes it capable of analyzing hundreds of metabolites simultaneously. Recently, some reports revealed the attempts to use it for metabolic identification and quantification related to some specific bio-functions [19–21]. HPLC-MS/MS was used for the analysis of bioactive ingredients responding to UV-B radiation in *D. officinale* [19]. HPLC-MS/MS was used for co-analysis between metabolites and anti-inflammatory activities in *D. chrysanthum* [25]. HPLC-MS/MS was used for the identification of polysaccharides that prevent ethanol-induced liver injury in *D. huoshanense* [26]. HPLC-MS/MS was used for co-analysis between polysaccharides and polycystic ovary syndrome in *D. nobile* [27]. HPLC-MS/MS was used for co-analysis between metabolites and diabetic myocardial fibrosis in *D. officinale* [28]. HPLC-MS/MS was used for co-analysis between metabolites and suppression rates in A549 lung cancer cells in *D. nobile* [29]. HPLC-MS/MS was used for the comparison of chemicals related to antioxidant activities between *D. huoshanense* and *D. officinale* [20]. HPLC-MS/MS was used for identification of antioxidant compounds in *D. catenatum* flower [12]. Here, HPLC-MS/MS was used for identification of the chemical basis related to antioxidant activities in vitro in *D. nobile* flower. Furthermore, the relative quantification results by HPLC-MS/MS were verified by the same common detection methods. HPLC-MS/MS would also be widely used for metabolic identification and quantification in chemical-function analysis in plants [30].

### 3.8. Some Enriched Flavonoids and Organic Acids Formed the Main Antioxidant Basis of the *D*. *nobile* Flower

ABTS scavenging, DPPH scavenging, and ferric reduction were generally used to evaluate in-vitro antioxidant activities [9, 12]. The extracts from flower of *D. nobile* showed significant higher ABTS scavenging rates, DPPH scavenging rates, and ferric-reducing power than those from root, stem, leaf, and fruit in this paper. The flower extracts of *D. officinale*, *D. sabin*, *D. devonianum*, and *D. catenatum* had also been reported to possess relatively high antioxidant activities [9, 11–13]. But the antioxidant activities related chemical basis was poorly studied in *Dendrobium* flower. Polysaccharides in the flowers of *D. devonianum* have been reported to be correlated with its antioxidant activities [11]. Phenolic glycosides in the methanolic extract of the flower were identified as antioxidant components in *D. catenatum* [12]. Here, 72 compounds mainly belong to three classes of metabolites amino acid and its derivatives, organic acid and its derivatives, and flavonoids were correlated to the higher antioxidant activities of flower in *D. nobile*. Furthermore, eight components of rutin, astragalin, isomucronulatol-7-O-glucoside, quercetin 4′-O-glucoside, methylquercetin O-hexoside, p-coumaric acid, caffeic acid and caffeic acid O-glucoside were identified to play a key contribution to antioxidant activities in vitro. Quercetin extracted from *D. officinale* showed antioxidant effect to UV-B exposure [19, 21]. The major compounds contributed to the antioxidative activities were identified as 1-O-caffeoyl-*β*-D-glucoside, rutin, and isoquercitrin in *D. catenatum* [12]. The antioxidant activities of *D. huoshanense* were also mainly attributed to its high content of flavonoids [20]. The novel finding of antioxidative flavonoids and organic acids further enriched acknowledge about the antioxidant basis of *Dendrobium* flower. This will be helpful in the production of related healthy or beauty products, such as flower-tea, flower-wine, flower-biscuits, flower-mask, flower-cream, flower-toothpaste, and flower-capsules [1, 16, 21].

## 4. Conclusions

This paper firstly confirmed the best in-vitro antioxidant activities of *D. noblie* flower. A total of seventy-two metabolites were identified to be corresponded to antioxidant activities in vitro. Eight flavonoids and organic acids formed the key antioxidant basis of *D. nobile* flower. The quantification results of HPLC-MS/MS were also verified by the common methods. These results suggest that HPLC-MS/MS is suitable for quantitative chemical-function analysis in *D. nobile*.

## Figures and Tables

**Figure 1:** Comparison of antioxidant activities among the extracts from root, stem, leaf, flower, and fruit of *D. nobile*. (a) ABTS scavenging rate under different concentration of extracts. (b) DPPH scavenging rate under different concentration of extracts. (c) Ferric-reducing power under different concentration of extracts. Vitamin C was used as a positive control. ^∗^indicates *p* < 0.05, ^∗∗^indicates *p* < 0.01, when compared flower to root, stem, leaf, or fruit.

**Figure 2:** HPLC-MS/MS total ion chromatograms of extracts from flower of *D. nobile*. (a) Positive ion mode. (b) Negative ion mode.

**Figure 3:** Distribution of the detected metabolites in flower of *D. nobile*. (a) Flower of *D. nobile*. (b) The detected metabolites were classified into 11 kinds of chemical compounds (*n* = 712).

**Figure 4:** Significantly highly accumulated metabolites in flower compared to root, stem, leaf, and fruit. Each of Log_2_ (Flower/Root), Log_2_ (Flower/Stem), Log_2_ (Flower/Leaf), Log_2_ (Flower/Fruit) of the 46 components were more than 2.

**Figure 5:** Distribution of antioxidant activities associated metabolites in flower of *D. nobile*. (a) Relative distribution in flower (*n* = 72). (b) Proportion in flower compared to root, stem, leaf, and fruit. CSCF/CSCA the contents of one specific component in flower to the contents of this component in all of root, stem, leaf, flower, and fruit.

**Figure 6:** Detailed distribution of antioxidant activities associated metabolites in flower of *D. nobile*. (a) Antioxidant activities associated amino acid and its derivatives (*n* = 13). (b) Antioxidant activities associated organic acid and its derivatives (*n* = 11). (c) Antioxidant activities associated flavonoids (*n* = 20).

**Figure 7:** Detailed Proportion of antioxidant activities associated metabolites in flower compared to root, stem, leaf, and fruit. (a) Antioxidant activities associated amino acid and its derivatives. (b) Antioxidant activities associated organic acid and its derivatives. (c) Antioxidant activities associated flavonoids. CSCF/CSCA the contents of one specific component in flower to the contents of this component in all of root, stem, leaf, flower, and fruit.

**Figure 8:** Diagram for antioxidant basis of *D. nobile* flower. ^*a*^*p* < 0.01, more than 5% of relative distribution in antioxidant activities associated metabolites in flower of *D*. *nobile*, and more than 80% of CSCF/CSCA in flower compared to root, stem, leaf, and fruit ^*b*^*p* < 0.05.

**Figure 9:** Comparison of the detected results by HPLC-MS/MS and common determination method in *D*. *nobile*. (a) Amino acid and its derivatives (*n* = 123), (b) organic acid and its derivatives (*n* = 105), (c) flavonoids (*n* = 111), (d) total proteins, (e) total organic acids, (f) total flavonoids. (a), (b), and (c) were based on the results of HPLC-MS/MS. (d), (e), and (f) were detected by corresponded colorimetry or titrimetry.

**Table 1:** Correlation of antioxidant activities to metabolites in D. nobile.

NO.	Name	ABTS scavenging					DPPH scavenging					Ferric reducing					CSCF/TCCF (%)	CSCF/CSCA (%)
		100	200	500	1000	2000	100	200	500	1000	2000	100	200	500	1000	2000		
1	DTFC-HBA	0.900^∗^	0.937^∗^	0.819	0.488	0.533	0.963^∗∗^	0.939^∗^	0.923^∗^	0.666	0.496	0.607	0.766	0.797	0.864	0.894^∗^	0.0023	45.82
2	1-aminocyclopentanecarboxylate	0.860	0.941^∗^	0.798	0.728	0.656	0.889^∗^	0.829	0.817	0.810	0.536	0.597	0.734	0.717	0.894^∗^	0.846	0.0273	41.75
3	2-amino-1,3,4-tetradecanetriol	0.906^∗^	0.829	0.892^∗^	0.547	0.636	0.722	0.944^∗^	0.932^∗^	0.654	0.435	0.799	0.856	0.892^∗^	0.838	0.902^∗^	0.0004	24.19
4	2′-deoxycytidine 5′-diphosphate	0.865	0.906^∗^	0.774	0.414	0.495	0.960^∗∗^	0.912^∗^	0.891^∗^	0.602	0.446	0.569	0.738	0.773	0.830	0.867	0.0440	55.39
5	2-hydroxy-6-aminopurine	0.848	0.947^∗^	0.778	0.680	0.528	0.936^∗^	0.833	0.838	0.818	0.645	0.506	0.658	0.651	0.848	0.810	0.0732	31.79
6	2-methylglutaric acid	0.888^∗^	0.962^∗∗^	0.803	0.554	0.511	0.991^∗∗^	0.908^∗^	0.902^∗^	0.733	0.578	0.546	0.715	0.733	0.863	0.866	0.0432	54.54
7	3-hydroxybutyrate	0.764	0.856	0.647	0.383	0.542	0.943^∗^	0.783	0.736	0.514	0.267	0.487	0.688	0.699	0.808	0.800	0.0135	42.96
8	5-aminosalicylic acid	0.852	0.946^∗^	0.758	0.541	0.500	0.991^∗∗^	0.865	0.855	0.712	0.548	0.501	0.681	0.692	0.845	0.835	0.1050	69.70
9	5-oxoproline	0.759	0.864	0.644	0.422	0.529	0.945^∗^	0.769	0.729	0.553	0.317	0.462	0.663	0.668	0.805	0.785	0.0054	48.62
10	6-aminohexanoic acid	0.821	0.916^∗^	0.715	0.446	0.451	0.998^∗∗^	0.849	0.834	0.635	0.494	0.462	0.656	0.676	0.810	0.813	0.0087	51.43
11	8-gingerol	0.837	0.934^∗^	0.740	0.502	0.445	0.998^∗∗^	0.858	0.853	0.694	0.569	0.462	0.648	0.664	0.816	0.813	0.0077	62.04
12	8-oxo-dGMP	0.769	0.820	0.658	0.330	0.613	0.888^∗^	0.798	0.733	0.434	0.129	0.575	0.761	0.779	0.820	0.832	0.0003	36.85
13	9(S)-HpOTrE	0.860	0.867	0.778	0.378	0.539	0.902^∗^	0.913^∗^	0.882^∗^	0.543	0.351	0.629	0.781	0.821	0.826	0.878	0.0009	56.95
14	Adipic acid	0.880^∗^	0.956^∗^	0.791	0.539	0.507	0.993^∗∗^	0.901^∗^	0.892^∗^	0.719	0.562	0.536	0.710	0.727	0.858	0.861	0.0533	57.13
15	*α*-ketoglutaric acid	0.803	0.872	0.695	0.334	0.418	0.974^∗∗^	0.855	0.832	0.538	0.416	0.470	0.663	0.699	0.775	0.807	0.0050	65.87
16	Angelol-K	0.837	0.939^∗^	0.771	0.671	0.450	0.936^∗^	0.828	0.848	0.838	0.731	0.458	0.606	0.604	0.809	0.779	0.0378	27.11
17	Astragalin	0.858	0.906^∗^	0.766	0.412	0.466	0.967^∗∗^	0.906^∗^	0.890^∗^	0.609	0.476	0.542	0.715	0.750	0.817	0.853	0.8209	96.06
18	Caffeic acid	0.859	0.903^∗^	0.768	0.407	0.477	0.962^∗∗^	0.907^∗^	0.889^∗^	0.600	0.457	0.553	0.724	0.760	0.820	0.858	1.3346	91.91
19	Caffeic acid O-glucoside	0.821	0.878	0.728	0.367	0.370	0.961^∗∗^	0.877	0.873	0.593	0.527	0.468	0.643	0.684	0.759	0.801	0.3282	85.94
20	Calycosin-7-O-glucoside	0.837	0.861	0.743	0.345	0.517	0.920^∗^	0.891^∗^	0.856	0.515	0.327	0.588	0.756	0.795	0.813	0.860	0.0050	44.83
21	Cyanidin 3-O-glucoside	0.851	0.909^∗^	0.758	0.415	0.443	0.976^∗∗^	0.898^∗^	0.886^∗^	0.620	0.502	0.517	0.693	0.727	0.808	0.840	0.0366	87.84
22	Cyanidin O-acetylhexoside	0.854	0.902^∗^	0.761	0.402	0.472	0.966^∗∗^	0.902^∗^	0.883^∗^	0.596	0.455	0.544	0.718	0.754	0.817	0.853	0.0509	94.00
23	*δ*-Aminolevulinic acid-HCL	0.845	0.928^∗^	0.745	0.463	0.471	0.997^∗∗^	0.875	0.860	0.652	0.506	0.495	0.682	0.704	0.827	0.835	0.0434	53.72
24	D-glutamine	0.880^∗^	0.957^∗^	0.791	0.545	0.520	0.992^∗∗^	0.898^∗^	0.888^∗^	0.718	0.550	0.542	0.716	0.731	0.864	0.864	4.7157	60.99
25	Diethanolamine	0.867	0.942^∗^	0.817	0.779	0.652	0.866	0.830	0.827	0.858	0.597	0.605	0.726	0.706	0.891^∗^	0.840	0.0179	37.61
26	Diosgenin	0.874	0.914^∗^	0.784	0.431	0.513	0.961^∗∗^	0.918^∗^	0.897^∗^	0.613	0.446	0.582	0.750	0.783	0.842	0.876	0.1529	46.12
27	DL-pecolinic acid	0.872	0.943^∗^	0.800	0.678	0.693	0.904^∗^	0.850	0.823	0.756	0.448	0.633	0.780	0.768	0.916^∗^	0.878	3.2369	41.35
28	D-norvaline	0.840	0.930^∗^	0.739	0.498	0.527	0.986^∗∗^	0.856	0.833	0.657	0.461	0.513	0.701	0.713	0.848	0.841	2.2341	50.51
29	dUDP	0.863	0.907^∗^	0.771	0.414	0.488	0.963^∗∗^	0.910^∗^	0.890^∗^	0.603	0.452	0.561	0.732	0.766	0.827	0.863	0.0435	56.10
30	Hesperetin 5-O-glucoside	0.825	0.881^∗^	0.730	0.366	0.392	0.964^∗∗^	0.880^∗^	0.871	0.586	0.501	0.482	0.659	0.698	0.770	0.811	0.0778	85.24
31	Hesperidin	0.844	0.892^∗^	0.751	0.386	0.438	0.962^∗∗^	0.896^∗^	0.882^∗^	0.592	0.476	0.522	0.695	0.734	0.797	0.837	0.0674	92.29
32	Isomucronulatol-7-O-glucoside	0.822	0.877	0.730	0.366	0.375	0.960^∗∗^	0.879^∗^	0.873	0.590	0.520	0.473	0.647	0.689	0.761	0.804	0.7168	87.56
33	Kaji-ichigoside F1	0.847	0.892^∗^	0.753	0.384	0.462	0.960^∗∗^	0.898^∗^	0.878^∗^	0.581	0.445	0.538	0.712	0.749	0.808	0.847	0.0218	91.17
34	Levodopa	0.844	0.894^∗^	0.748	0.384	0.457	0.965^∗∗^	0.895^∗^	0.875	0.583	0.449	0.530	0.706	0.743	0.806	0.843	0.1576	80.70
35	L-isoleucine	0.827	0.919^∗^	0.724	0.445	0.439	0.999^∗∗^	0.858	0.846	0.642	0.515	0.463	0.654	0.677	0.807	0.814	5.2740	53.18
36	L-leucine	0.827	0.920^∗^	0.724	0.449	0.442	0.999^∗∗^	0.858	0.845	0.644	0.515	0.463	0.655	0.676	0.809	0.815	7.7092	53.34
37	L-serine	0.874	0.949^∗^	0.818	0.753	0.662	0.885^∗^	0.842	0.833	0.834	0.563	0.613	0.743	0.726	0.902^∗^	0.855	0.1720	37.96
38	L-tyrosine	0.843	0.914^∗^	0.750	0.434	0.405	0.986^∗∗^	0.886^∗^	0.883^∗^	0.651	0.564	0.477	0.655	0.687	0.793	0.819	0.0469	74.40
39	L-valine	0.845	0.933^∗^	0.744	0.493	0.518	0.990^∗∗^	0.864	0.843	0.659	0.473	0.514	0.701	0.715	0.847	0.843	0.0953	52.93
40	Methylenesuccinic acid	0.874	0.963^∗∗^	0.799	0.656	0.562	0.957^∗^	0.867	0.863	0.796	0.600	0.547	0.704	0.703	0.876	0.848	0.0004	39.37
41	methylQuercetin O-hexoside	0.838	0.888^∗^	0.744	0.378	0.427	0.962^∗∗^	0.891^∗^	0.878	0.586	0.477	0.512	0.687	0.725	0.790	0.830	0.4173	90.99
42	N2-methylguanosine	0.790	0.842	0.680	0.292	0.477	0.939^∗^	0.844	0.803	0.468	0.287	0.516	0.706	0.742	0.783	0.820	0.0039	42.74
43	N7-methylguanosine	0.817	0.895^∗^	0.715	0.386	0.392	0.989^∗∗^	0.864	0.854	0.603	0.512	0.451	0.640	0.673	0.777	0.802	0.0088	52.97
44	N-acetyl-D-glucosamine	0.834	0.920^∗^	0.734	0.513	0.588	0.961^∗∗^	0.841	0.808	0.641	0.391	0.547	0.730	0.736	0.866	0.850	0.0017	49.51
45	N-acetylglycine	0.849	0.938^∗^	0.752	0.497	0.474	0.998^∗∗^	0.872	0.862	0.683	0.538	0.492	0.676	0.694	0.832	0.833	0.0018	64.55
46	Naringin	0.826	0.933^∗^	0.734	0.541	0.427	0.988^∗∗^	0.839	0.842	0.732	0.623	0.436	0.616	0.628	0.804	0.791	0.0015	56.10
47	Neocryptotanshinone	0.876	0.915^∗^	0.792	0.441	0.479	0.959^∗∗^	0.923^∗^	0.911^∗^	0.637	0.503	0.568	0.730	0.765	0.828	0.866	0.0040	52.11
48	p-Coumaric acid	0.857	0.901^∗^	0.764	0.402	0.476	0.962^∗∗^	0.906^∗^	0.886^∗^	0.596	0.453	0.551	0.723	0.759	0.818	0.856	0.6013	87.50
49	Phellodenol H O-hexoside	0.848	0.883^∗^	0.752	0.375	0.527	0.942^∗^	0.896^∗^	0.862	0.544	0.351	0.584	0.757	0.792	0.830	0.868	0.0092	63.80
50	Phenylacetylglutamine	0.889^∗^	0.943^∗^	0.801	0.491	0.533	0.980^∗∗^	0.922^∗^	0.904^∗^	0.667	0.490	0.582	0.752	0.777	0.866	0.885^∗^	0.0517	73.27
51	Pipecolic acid	0.846	0.928^∗^	0.779	0.706	0.668	0.882^∗^	0.815	0.796	0.779	0.487	0.596	0.737	0.719	0.892^∗^	0.842	0.6891	41.01
52	Plantagoside	0.904^∗^	0.945^∗^	0.824	0.504	0.538	0.968^∗∗^	0.940^∗^	0.925^∗^	0.680	0.509	0.607	0.767	0.795	0.870	0.896^∗^	0.0054	76.21
53	Polygalaxanthone VII	0.859	0.892^∗^	0.768	0.393	0.499	0.946^∗^	0.909^∗^	0.885^∗^	0.577	0.415	0.577	0.744	0.781	0.824	0.866	0.0233	82.41
54	Purine	0.793	0.912^∗^	0.699	0.559	0.470	0.960^∗∗^	0.790	0.783	0.715	0.556	0.429	0.611	0.610	0.804	0.771	0.0117	56.54
55	Quercetin	0.828	0.883^∗^	0.736	0.375	0.386	0.963^∗∗^	0.883^∗^	0.877	0.597	0.521	0.481	0.655	0.695	0.769	0.810	0.0168	82.59
56	Quercetin 4′-O-glucoside	0.821	0.879^∗^	0.727	0.369	0.369	0.964^∗∗^	0.876	0.872	0.596	0.531	0.465	0.640	0.681	0.759	0.800	0.6651	85.22
57	Quercetin 5-O-hexoside	0.826	0.881^∗^	0.732	0.370	0.385	0.963^∗∗^	0.881^∗^	0.874	0.591	0.514	0.479	0.654	0.695	0.768	0.809	0.0771	83.09
58	Quercetin O-malonylhexoside	0.841	0.881^∗^	0.749	0.369	0.442	0.950^∗^	0.896^∗^	0.879^∗^	0.572	0.452	0.533	0.703	0.743	0.793	0.838	0.0223	75.85
59	Quercetin-O-glucoside	0.834	0.890^∗^	0.734	0.372	0.449	0.970^∗∗^	0.884^∗^	0.863	0.571	0.438	0.514	0.696	0.732	0.800	0.835	0.0355	79.23
60	Quercitrin	0.861	0.890^∗^	0.767	0.425	0.637	0.920^∗^	0.893^∗^	0.844	0.548	0.266	0.653	0.819	0.843	0.878	0.901^∗^	0.0070	52.83
61	Rhodomyrtone	0.876	0.912^∗^	0.788	0.430	0.511	0.956^∗^	0.921^∗^	0.901^∗^	0.613	0.450	0.587	0.752	0.786	0.840	0.877	0.0487	39.16
62	Rutin	0.852	0.898^∗^	0.760	0.399	0.451	0.963^∗∗^	0.902^∗^	0.887^∗^	0.601	0.478	0.533	0.705	0.742	0.806	0.845	2.4000	96.16
63	Scopolamine	0.809	0.855	0.708	0.314	0.422	0.946^∗^	0.868	0.845	0.518	0.397	0.501	0.682	0.724	0.769	0.815	0.0702	80.18
64	Sibiricose A6	0.834	0.930^∗^	0.738	0.492	0.420	0.998^∗∗^	0.860	0.859	0.695	0.592	0.450	0.634	0.654	0.804	0.805	0.0016	55.05
65	Sibirioside A	0.827	0.881^∗^	0.724	0.355	0.465	0.964^∗∗^	0.877	0.850	0.547	0.395	0.521	0.705	0.741	0.802	0.836	0.0122	81.31
66	Threonyl carbamoyl adenosine	0.899^∗^	0.976^∗∗^	0.828	0.669	0.580	0.960^∗∗^	0.894^∗^	0.891^∗^	0.809	0.609	0.580	0.732	0.733	0.894^∗^	0.872	0.0039	39.87
67	Tiliroside	0.822	0.875	0.729	0.361	0.377	0.957^∗^	0.879^∗^	0.873	0.585	0.514	0.476	0.650	0.691	0.760	0.804	0.1808	87.70
68	trans-3-hydroxy-L-proline	0.803	0.899^∗^	0.694	0.461	0.539	0.967^∗∗^	0.815	0.782	0.603	0.378	0.496	0.690	0.699	0.833	0.819	0.0223	52.76
69	Tricetin O-hexoside	0.832	0.885^∗^	0.740	0.377	0.397	0.961^∗∗^	0.887^∗^	0.879^∗^	0.596	0.512	0.491	0.664	0.704	0.775	0.816	0.0664	82.69
70	Trifolin	0.851	0.910^∗^	0.757	0.417	0.443	0.979^∗∗^	0.897^∗^	0.885^∗^	0.622	0.504	0.514	0.691	0.725	0.809	0.840	0.0742	86.54
71	Vanillic acid	0.865	0.904^∗^	0.780	0.420	0.462	0.956^∗^	0.915^∗^	0.903^∗^	0.620	0.495	0.554	0.718	0.756	0.815	0.855	0.0085	86.75
72	Xanthosine	0.932^∗^	0.914^∗^	0.873	0.530	0.699	0.869	0.962^∗∗^	0.926^∗^	0.639	0.350	0.772	0.893^∗^	0.919^∗^	0.919^∗^	0.957^∗^	0.0054	42.84

CSCF/TCCF the contents of one specific component in flower to the total contents of 712 components in flower. CSCF/CSCA the contents of one specific component in flower to the contents of this component in all of root, stem, leaf, flower, and fruit. DTFC-HBA (2S, 3R)-2-{[{9-[(2R, 3R, 4S, 5R)-3,4-Dihydroxy-5-(hydroxymethyl)tetrahydro-2-furanyl]-9H-purin-6-yl}(methyl)carbamoyl]amino}-3-hydroxybutanoic acid, 9(S)-HpOTrE (9S, 10E, 12Z, 15Z)-9-Hydroperoxy-10, 12, 15-octadecatrienoate.

## Data Availability

All related data are included within the article.

## References

[1] Zheng S. G., Hu Y. D., Zhao R. X. (2018). Genome-wide researches and applications on dikendrobium. *Planta*.

[2] Mou Z., Zhao Y., Ye F. (2021). Identification, biological activities and biosynthetic pathway of dendrobium alkaloids. *Frontiers in Pharmacology*.

[3] Wang Y. H. (2021). Traditional uses and pharmacologically active constituents of dendrobium plants for dermatological disorders: a review. *Natural Products and Bioprospecting*.

[4] Zhang F., Shi J. S., Li D. D., Zheng C. Q. (2022). Potential neuroprotection by dendrobium nobile Lindl alkaloid in Alzheimer’s disease models. *Neural Regeneration Research*.

[5] Percário S., Da Silva Barbosa A., Varela E. L. P. (2020). Oxidative stress in parkinson’s disease: potential benefits of antioxidant supplementation. *Oxidative Medicine and Cellular Longevity*.

[6] Byrne N. J., Rajasekaran N. S., Abel E. D., Bugger H. (2021). Therapeutic potential of targeting oxidative stress in diabetic cardiomyopathy. *Free Radical Biology and Medicine*.

[7] Vatner S. F., Zhang J., Oydanich M., Berkman T., Naftalovich R., Vatner D. E. (2020). Healthful aging mediated by inhibition of oxidative stress. *Ageing Research Reviews*.

[8] Wang Y., Zhao J., Jiang L., Mu Y. (2021). The application of skin care product in melasma treatment. *Clinical, Cosmetic and Investigational Dermatology*.

[9] Abu F., Taib C. N. M., Moklas M. A. M., Akhir S. M. (2017). Antioxidant properties of crude extract, partition extract, and fermented medium of dendrobium sabin flower. *Evidence-Based Complementary and Alternative Medicine*.

[10] Zhang Y., Zhang L. H., Liu J. J., Liang J. L., Si J. P., Wu S. H. (2017). Dendrobium officinale leaves as a new antioxidant source. *Journal of Functional Foods*.

[11] Wang D., Fan B., Wang Y., Zhang L., Wang F. (2018). Optimum extraction, characterization, and antioxidant activities of polysaccharides from flowers of dendrobium devonianum. *International Journal of Analytical Chemistry*.

[12] Zhang X. F., Zhang S. J., Gao B. B. (2019). Identification and quantitative analysis of phenolic glycosides with antioxidant activity in methanolic extract of Dendrobium catenatum flowers and selection of quality control herb-markers. *Food Research International*.

[13] Li L. Z., Lei S. S., Li B. (2020). Dendrobium officinalis flower improves learning and reduces memory impairment by mediating antioxidant effect and balancing the release of neurotransmitters in senescent rats. *Combinatorial Chemistry & High Throughput Screening*.

[14] Warinhomhoun S., Muangnoi C., Buranasudja V. (2021). Antioxidant activities and protective effects of dendropachol, a new bisbibenzyl compound from dendrobium pachyglossum, on hydrogen peroxide-induced oxidative stress in HaCaT keratinocytes. *Antioxidants*.

[15] Wang J. H., Zhang B. W., Luo J. P. (2015). Molecular weight, chain conformation and antioxidant activities of sulfated beta-D-galactan derivatives from dendrobium nobile Lindl. *Current Topics in Nutraceutical Research*.

[16] Pisoschi A. M., Pop A., Cimpeanu C., Predoi G. (2016). Antioxidant capacity determination in plants and plant-derived products: a review. *Oxidative Medicine and Cellular Longevity*.

[17] Huang G., Mei X., Hu J. (2017). The antioxidant activities of natural polysaccharides. *Current Drug Targets*.

[18] Shen N., Wang T., Gan Q., Liu S., Wang L., Jin B. (2022). Plant flavonoids: classification, distribution, biosynthesis, and antioxidant activity. *Food Chemistry*.

[19] Chen Y., Shen Q., Lv P., Sun C. (2020). Comparative metabolomic analyses of Dendrobium officinale Kimura et Migo responding to UV-B radiation reveal variations in the metabolisms associated with its bioactive ingredients. *PeerJ*.

[20] Wan J., Gong X., Wang F. (2022). Comparative analysis of chemical constituents by HPLC-ESI-MS(n) and antioxidant activities of dendrobium huoshanense and dendrobium officinale. *Biomedical Chromatography*.

[21] Zhu Y., Yu J., Jiao C. (2019). Optimization of quercetin extraction method in dendrobium officinale by response surface methodology. *Heliyon*.

[22] Zhang Y., You S., Wang D. (2022). Fermented dendrobium officinale polysaccharides protect UVA-induced photoaging of human skin fibroblasts. *Food Sciences and Nutrition*.

[23] Wang L., Mao Y. G., Zeng X. (2022). Structure and bioactivities of a novel polysaccharide extracted from dendrobium huoshanense by subcritical water. *Frontiers in Nutrition*.

[24] Wang Y., Liao X., Zhou C. (2020). Identification of C-glycosyl flavones and quality assessment in dendrobium nobile. *Rapid Communications in Mass Spectrometry*.

[25] Yang L., Qin L. H., Bligh S. A. (2006). A new phenanthrene with a spirolactone from dendrobium chrysanthum and its anti-inflammatory activities. *Bioorganic & Medicinal Chemistry*.

[26] Wang X. Y., Luo J. P., Chen R., Zha X. Q., Pan L. H. (2015). Dendrobium huoshanense polysaccharide prevents ethanol-induced liver injury in mice by metabolomic analysis. *International Journal of Biological Macromolecules*.

[27] Zhang S., Tu H., Zhu J. (2020). Dendrobium nobile Lindl. polysaccharides improve follicular development in PCOS rats. *International Journal of Biological Macromolecules*.

[28] Zeng J., Li D., Li Z., Zhang J., Zhao X. (2020). Dendrobium officinale attenuates myocardial fibrosis via inhibiting EMT signaling pathway in HFD/STZ-induced diabetic mice. *Biological and Pharmaceutical Bulletin*.

[29] Zheng S., Hu Y., Zhao R. (2020). Quantitative assessment of secondary metabolites and cancer cell inhibiting activity by high performance liquid chromatography fingerprinting in Dendrobium nobile. *Journal of Chromatography B*.

[30] Lam Y., Ng T. B., Yao R. M. (2015). Evaluation of chemical constituents and important mechanism of pharmacological biology in Dendrobium plants. *Evidence-Based Complementary and Alternative Medicine*.

